The article "Research on the Evaluation Method of Enterprises' Independent Innovation Ability Based on Improved BP Neural Network and DQN Algorithm" was retracted in 2023. Reasons: unreliable results or conclusions; concerns about the data; concerns about the results or conclusions; concerns about the peer review.

# Research on the Evaluation Method of Enterprises' Independent Innovation Ability Based on Improved BP Neural Network and DQN Algorithm

**DOI:** 10.1155/2022/8250879

**Published:** 2022-03-24

**Authors:** Yipin Fan, Ding Ding, Hong Qin

**Affiliations:** ^1^College of Management, Ocean University of China, Qingdao, Shandong 266100, China; ^2^College of Foreign Languages, Shangqiu Normal University, Shangqiu, Henan 476000, China

## Abstract

The development of enterprises has a very important influence on promoting national economic growth and improving comprehensive economic strength. This work evaluates the independent innovation ability of enterprises, analyzes the characteristics and difficulties of technological innovation of enterprises, and proposes corresponding solutions to promote independent technological innovation of enterprises. Firstly, the characteristics of the research object are clarified, and on the basis of relevant research, the theory of technological innovation and evaluation at home and abroad is expounded. At the same time, the basic theory of the improved BP neural network and DQN algorithm is introduced, which provides a theoretical basis for the research of the thesis. Secondly, according to the characteristics of enterprise technological innovation, an index system for evaluating the technological innovation capability of enterprises is constructed. Then, according to the related theory of the improved BP neural network and DQN algorithm, a neural network model for evaluating the technological innovation capability of enterprises is designed, and the validity of the model is verified through empirical research. Finally, this paper applies the evaluation model to the surveyed enterprises, comprehensively analyzes the characteristics and existing problems of independent technological innovation of enterprises, and proposes practical and feasible countermeasures to improve technological innovation capabilities from the perspective of enterprises themselves. The research results of this paper can be used as an effective supplement to the research on independent technological innovation of enterprises, and at the same time promote the continuous improvement of independent technological innovation capabilities of enterprises.

## 1. Introduction

Innovation is the soul of a nation's progress and an inexhaustible driving force for the prosperity of a country. Technological innovation is the first driving force of economic growth, is the main source of national economic growth, and promotes the prosperity of the global economy. Among them, enterprise technological innovation is an important part of the national technological innovation system, and enterprises are the experimental grounds of national technological innovation, the bases of innovation achievement and industrialization, and at the same time it is the main body of innovation. The development of technology-based enterprises has a very important impact on promoting the economic growth of a country or region, enhancing market competitiveness, and improving overall economic strength. Technology-based enterprises have become an active force for the country to develop high-tech industries. Technology-based enterprises are the source of vitality for technological innovation, the foundation of the entire high-tech industry, the main force in achieving technological leapfrogging, and one of the important supports of the knowledge economy [1–7].

The article "Research on the Evaluation Method of Enterprises' Independent Innovation Ability Based on Improved BP Neural Network and DQN Algorithm" was retracted in 2023. Reasons: unreliable results or conclusions; concerns about the data; concerns about the results or conclusions; concerns about the peer review.

In today's economic globalization, the fiercely competitive market environment and ever-changing customer needs require technology companies to continuously carry out technological innovation. Continuous technological innovation is the soul of the development of technological enterprises [8–13]. The research significance of the thesis mainly has the following two aspects: (1) theoretical significance: the theory of science and technology enterprises is proposed and developed under the unique national conditions of our country, and the research on its special technological innovation mechanism has not yet formed a mature system. Based on the definition of the concept of technology-based enterprises and a summary of technological innovation capabilities, this paper innovatively constructs an evaluation index system for technology innovation capabilities of technology-based enterprises based on excellent performance based on the excellent performance evaluation model, and establishes an evaluation model. This is a useful supplement to the research on technological innovation of my country's technology-based enterprises, and it has enriched and perfected the technological innovation theory of my country's technology-based enterprises. At the same time, this paper applies the improved BP neural network and DQN algorithm related theories to construct a neural network evaluation model for evaluating the technological innovation capabilities of technology-based enterprises, which enriches the application of BP neural network. (2) Practical significance: technology-based enterprises are not only an effective carrier for accelerating the transformation of scientific and technological achievements and realizing technological innovation, but also an important source of national economic growth. The evaluation of technological innovation capabilities of technology-based enterprises, on the one hand, helps technology-based enterprise managers analyze their own technological innovation capabilities and determine development goals; on the other hand, they further summarize their technological innovation experience, strengthen technological innovation management, and improve Technological innovation mechanisms, adopting reasonable technological innovation strategies, increasing investment in technological innovation, and maintaining and improving competitiveness are all of great significance. Through questionnaire surveys and on-site interviews, this research deeply understands the true status quo of enterprise technological innovation capabilities, analyzes its characteristics and existing problems, and proposes specific improvement countermeasures and policy recommendations, which will promote the continuous improvement of technological innovation capabilities of technology-based enterprises Has important practical significance.

The article "Research on the Evaluation Method of Enterprises' Independent Innovation Ability Based on Improved BP Neural Network and DQN Algorithm" was retracted in 2023. Reasons: unreliable results or conclusions; concerns about the data; concerns about the results or conclusions; concerns about the peer review.

## 2. Related Work

Many scholars have not been satisfied with the definition of the meaning and structure of technological innovation capabilities in the research on the technological innovation capabilities of enterprises. The evaluation index system and evaluation model of technological innovation capability.

In foreign countries, Steele used a checklist to evaluate R&D activities. The specific content took into account innovation goals, markets, resource allocation, production processes, project sustainability, etc. [14]. Ransley and Rogers conducted a research summary on the best R&D practices of enterprises, and put forward 7 aspects that should be considered: technology strategy, project selection and management, core competence, effectiveness, external awareness, technology transfer and personnel, and use fuzzy Comprehensive evaluation analyzes and studies related aspects [15]. Based on innovative system integration and network model, Terziovski measures the organization's innovation ability from four aspects: innovation input, innovation process, innovative products and innovation strategy [16]. Richard constructed a model of the relationship between enterprise technological innovation capability and core competitiveness based on DEA evaluation method [17]. Wang et al., in the study of “Evaluating Enterprise Technological Innovation Ability Based on Uncertain Conditions,” constructed the hierarchical structure model of technological innovation ability of high-tech enterprises, and adopted the nonlinear fuzzy integral method to evaluate the technological innovation ability of enterprises. Empirical et al. research proves that this method plays an important role in the evaluation of technological innovation capabilities of high-tech enterprises [18].

The article "Research on the Evaluation Method of Enterprises' Independent Innovation Ability Based on Improved BP Neural Network and DQN Algorithm" was retracted in 2023. Reasons: unreliable results or conclusions; concerns about the data; concerns about the results or conclusions; concerns about the peer review.

There are also many domestic researches on the evaluation of technological innovation capabilities. The main research results are Xu et al. discussed the general procedure of the evaluation of enterprise technological innovation capabilities and the general process of solving practical problems based on the mathematical model of fuzzy comprehensive evaluation, in order to make the evaluation of enterprise technological innovation capability is more scientific, standardized and quantitative [19]. Lu and Han used the close value method to evaluate the technological innovation capabilities of enterprises, and to a certain extent overcomes the large amount of calculation and evaluation indicators that exist in the use of analytic hierarchy process, efficiency coefficient method, gray theory, fuzzy mathematics and other methods for multiobjective evaluation. The determination of weight lacks theoretical basis and other shortcomings [20]. Su and Zhang used the artificial neural network model based on BP algorithm to evaluate the technological innovation ability of enterprises, and opened up a new method for the evaluation of enterprise innovation ability [21]. Lu et al. proposed a secondary relative evaluation method to measure the technological innovation capabilities of enterprises. This method first uses the analytic hierarchy process (AHP) to measure the comprehensive index status, and then uses the BCC model in the data envelopment analysis (DEA) method to measure the secondary Relative evaluation value, this method eliminates the influence of the quality of objective basic conditions, and thus more accurately reflects the role of people's effective subjective efforts in enhancing the technological innovation capabilities of enterprises [22]. Based on the innovation chain model proposed by Kline and Rosenberg, Dai et al. selected 10 indicators from four aspects, including technology accumulation, R&D investment, production and digestion of new technologies, and sales of new products, as the evaluation index system for enterprise technological innovation capabilities. Use index method and comprehensive index evaluation method to evaluate [23]. Zhu et al. used the mean-variance model, also referred to as the EV model, to put forward a method to evaluate the technological innovation capabilities of enterprises, and apply the Lagrangian multiplier method to solve the weight coefficients of various indicators, for scientific evaluation and timely adjustment of enterprise technological innovation The strategy provides the basis [24].

The research contributions of the paper are as follows:

1. This work evaluates the independent innovation ability of enterprises, analyzes the characteristics and difficulties of technological innovation of enterprises, and proposes corresponding solutions to promote independent technological innovation of enterprises
2. The basic theory of improved BP neural network and DQN algorithm is introduced
3. A neural network model is designed to evaluate the technological innovation capability of enterprises, and the validity of the model is verified through empirical research

The article "Research on the Evaluation Method of Enterprises' Independent Innovation Ability Based on Improved BP Neural Network and DQN Algorithm" was retracted in 2023. Reasons: unreliable results or conclusions; concerns about the data; concerns about the results or conclusions; concerns about the peer review.

## 3. Method

The independent innovation capability of an enterprise is a nonlinear system. Quantitative analysis of complex enterprises involves many influencing factors, identifying the hidden layer between targets and indicators of various factors, and the artificial neural network method is a way to solve nonlinear and complex problems. The systematic and more effective method can be better applied to the evaluation research of the independent innovation ability of high-tech enterprises. Based on combing and summarizing the related theoretical research of high-tech independent innovation capabilities, this paper will combine high-tech independent innovation capabilities, improved BP network and DQN algorithm research methods, and combined with MATLAB software for calculation and simulation. Realize the research methods combine theoretical research with empirical research, and combine qualitative analysis with quantitative analysis. The technical roadmap is shown in Figure 1. The research roadmap in Figure 1 is the combined use of the BP neural network algorithm and the DQN algorithm, and the advantages of the two algorithms are used to analyze the data, so as to conduct more analysis on the data.

### 3.1. BP Neural Network and Improved Model

#### 3.1.1. Characteristics of BP Neural Network

Artificial neural networks have attracted great attention in recent years, especially the multilayer feedforward network based on error back propagation algorithm, which can approximate any continuous function with arbitrary precision. The BP network is shown in Figure 2.

It has the following outstanding advantages in the evaluation of the core competitiveness of high-tech enterprises: (1) The error is small and the stability is good. The artificial neural network model can make the system error meet any accuracy requirements through continuous learning and training samples. The network can fully approximate arbitrarily complex nonlinear functions with convergence. At the same time, the network composed of threshold neurons has better performance and can improve fault tolerance and storage capacity, so it has strong robustness and fault tolerance. In addition, the neural network does not have harsh requirements and restrictions on the distribution and covariance of the samples, and the artificial neural network is not very sensitive to noise data and has strong robustness. (2) Strong adaptability. The artificial neural network has the ability of self-adaptation, self-organization and self-learning, and can adapt to the changes of training samples. When the training sample adds new data, the neural network can adjust itself according to the new data, so as to enable the mapping relationship of the representation Can better describe new samples. And with the increase of samples and the advancement of time, the network can implement dynamic tracking and evaluation according to actual changes. When processing information, the nonlinear dynamic system itself is constantly changing to learn and adapt to unknown or uncertain systems. (3) Good practicability. The network can also process quantitative and qualitative information at the same time. All quantitative or qualitative information is equipotentially distributed and stored in each neuron in the network; the artificial neural network selects the network model structure of the sample to be evaluated and evaluates the core competitiveness of the enterprise The optimal algorithm criterion of the algorithm is repeatedly trained, and the network structure is continuously adjusted and optimized until stability is reached, and the data is evaluated and sorted by the model, thereby ensuring the objectivity and practicability of the evaluation structure and evaluation results. It can better obtain the objective mapping relationship through the learning of samples, and will not affect the accuracy of evaluation due to the intervention of more subjective factors. (4) It can handle nonlinear problems well. Because network neurons have two different states of activation or inhibition, this behavior is manifested as a nonlinear relationship. Therefore, when processing nonlinear data, the accuracy of artificial neural networks is significantly higher than other evaluation methods.

The article "Research on the Evaluation Method of Enterprises' Independent Innovation Ability Based on Improved BP Neural Network and DQN Algorithm" was retracted in 2023. Reasons: unreliable results or conclusions; concerns about the data; concerns about the results or conclusions; concerns about the peer review.

#### 3.1.2. Improvement of LM Algorithm of BP Neural Network

Due to the three-layer perceptron and nonlinear optimization capabilities of the BP network, its calculation can approximate any nonlinear function with arbitrary precision, so this algorithm has been widely developed and applied, but in practical applications, the BP network also has shortcomings and the areas that need improvement: (1) The number of training times is large, and the convergence speed is slow. The BP network algorithm also requires thousands of times of learning and training to achieve convergence for a common problem. The training time may be slow for some complex problems and very long. Because the minimization objective function of the gradient descent method is very complicated, the zigzag image will inevitably appear and the BP algorithm will be inefficient. To solve this problem, the methods to improve the convergence speed of the network include increasing the momentum term, improving the error function, adaptively adjusting the learning rate, and introducing the steepness factor. (2) It is easy to fall into the local minimum and cannot guarantee the global optimal. Because the BP learning algorithm uses the gradient descent method, the connection weight space is not only a parabola with a minimum point, but also a hypersurface with multiple minimum points. The training starts from a certain starting point and reaches the minimum value of the error along the slope of the error function, so different starting points may result in different minimum values and no optimal solution. If the number of network layers and neurons are increased in order to improve the accuracy of the training results, the network complexity will inevitably increase and the network training time will be increased.

There are also many researches on the improvement of BP network. At present, the more commonly used optimization algorithms include additional momentum algorithm, variable rate algorithm, adaptive learning rate method, RPROP method, conjugate gradient algorithm, and Gaussian. Newton's algorithm, Levenbel-g. Marquardt algorithm, etc.; and the LM algorithm is the method with the fastest convergence speed and the best robustness among the above algorithms. This article uses the LM optimization algorithm to optimize the BP neural network.

In Newton's algorithm, when the Hessian matrix is not positive definite, the Newton direction may point to a local pole, and the Hessian matrix can be changed to positive definite by adding a positive definite matrix to the Hessian matrix. The LM algorithm is a combination of the gradient descent method and the Gauss–Newton method. It also has Gaussian. The local convergence characteristics of the Newton method and the global characteristics of the gradient descent method; the LM algorithm converges much faster than the gradient method, and the algorithm is relatively stable.

In BP network, the loss function is calculated as follows:

(1) $$\begin{array}{c} E\left(x\right)=\frac{1}{2}\sum_{i=1}^{n}{\left[d\left(i\right)-y\left(i\right)\right]}^{2}. \end{array}$$

Through backpropagation, the updated weight is

(2) $$\begin{array}{c} x^{\left(k+1\right)}=x^{\left(k\right)}+\Delta x. \end{array}$$

For Newton's algorithm,

(3) $$\begin{array}{c} \Delta x=-\frac{\nabla E\left(x\right)}{\nabla^{2}E\left(x\right)}. \end{array}$$

In order to make Hessian matrices all invertible, it is necessary to approximate them:

(4) $$\begin{array}{c} \nabla E\left(x\right)=J^{T}\left(x\right)e\left(x\right), \end{array}$$

where *J*(*x*) is Jacobian matrix.

The article "Research on the Evaluation Method of Enterprises' Independent Innovation Ability Based on Improved BP Neural Network and DQN Algorithm" was retracted in 2023. Reasons: unreliable results or conclusions; concerns about the data; concerns about the results or conclusions; concerns about the peer review.

The LM algorithm improves the Gauss–Newton method, and the improved weight and threshold adjustment rule is

(5) $$\begin{array}{c} \Delta x=-{\left[J^{T}\left(x\right)J\left(x\right)+\mu I\right]}^{-1}J\left(x\right)E\left(x\right). \end{array}$$

Practice has proved that using the LM algorithm for network calculations can be many times faster than the gradient descent method. The LM optimization method has a fast learning speed and can achieve very good results in practical applications.

### 3.2. DQN Algorithm

Reinforcement learning algorithms can be divided into three categories: value based, policy based and actor critic. The most common one is the value based algorithm represented by DQN. This algorithm has only one value function network, no policy network, and actor-critic algorithm represented by DDPG and TRPO. This algorithm has both value function networks and there is a policy network.

The DQN algorithm is a method that uses stochastic gradient descent to update parameters in combination with neural networks, and then approximates the action state value function *Q*(*s*, *a*) as shown in Figure 3.

The problem of too large state space and action space can be handled by neural networks. The DQN algorithm uses the neural network structure to parameterize the state action value function *Q*(*s*, *a*), and combines it with the Q-Learning algorithm to avoid the large consumption of memory for data storage and the waste of time for data search. In the neural network of the DQN algorithm, the state *s* is used as the input value, and the neural network outputs the state action function value *Q*(*s*, *a*) corresponding to all actions *a* in this state. Then, according to the principle of *ε*-greedy, select the action a that can produce the largest *Q*(*s*, *a*) value to execute, or randomly select action a to execute.

The DQN algorithm can enable the agent to quickly optimize strategy *π* in the process of interacting with the environment. Existing research results show that in some games, the performance of the DQN algorithm can even greatly surpass that of humans. The reason why the DQN algorithm performs well is that the DQN algorithm uses two methods of experience playback and fixed target in the process of neural network parameter update. Experience replay refers to the memory bank set up for learning previous experiences in the process of interaction between the agent and the environment by the DQN algorithm. As an offline learning method, Q-Learning can not only learn current experiences, but also historical experiences, and even learn from other people's experiences. In this way, when the DQN algorithm performs parameter update, the experience is randomly selected from the memory bank for learning, which can disrupt the correlation between experiences and make the neural network update more efficient. In addition to experience playback, another method of fixing the target is also to disrupt relevance and improve learning efficiency. The DQN algorithm uses a fixed target and requires two neural networks with the same structure but different parameters. One of the two neural networks in the DQN algorithm is used to generate *Q* reality and the other is used to generate *Q* estimates. The neural network that generates the *Q* estimate has the latest parameters, while the neural network that generates the *Q* reality uses the old parameters, and the old parameters will be updated periodically according to the settings.

The article "Research on the Evaluation Method of Enterprises' Independent Innovation Ability Based on Improved BP Neural Network and DQN Algorithm" was retracted in 2023. Reasons: unreliable results or conclusions; concerns about the data; concerns about the results or conclusions; concerns about the peer review.

With the two methods of experience replay and fixed target, the agent can improve the strategy *π* more stably and efficiently during the learning process with DQN. The BP neural network algorithm has the characteristics of strong learning ability, and the DQN algorithm has the advantage of a wide range of learning. The combination of the two can better analyze and learn the data in a unified manner.

## 4. Experiments and Discussion

### 4.1. Survey Data

This survey was organized by the Development Planning Division of a provincial Science and Technology Department. The survey objects were technology-based enterprises funded by innovation funds. The survey content mainly included five aspects: basic company information, innovation resources, innovation process, innovation output, and innovation environment, use the form to conduct the survey. A total of 120 valid questionnaires were collected in this survey, and the data was classified and summarized. See Table 1 for the distribution of enterprise technology fields. In terms of the distribution of technical fields, the four fields of opto-mechanical and electronic integration, new materials, electronic information, and biomedicine account for 90.18%. This shows the general distribution characteristics of the industry of science and technology small and medium-sized enterprises in Hunan Province.

### 4.2. Training Loss and Testing Error

After the network is trained for 4000 steps, the training error reaches the expected error, and the convergence effect of the network is good, as shown in Figure 4.

The error between the predicted value and the actual value of the test sample is shown in Figure 5.

The article "Research on the Evaluation Method of Enterprises' Independent Innovation Ability Based on Improved BP Neural Network and DQN Algorithm" was retracted in 2023. Reasons: unreliable results or conclusions; concerns about the data; concerns about the results or conclusions; concerns about the peer review.

### 4.3. Evaluation Result Analysis

The neural network evaluation model established in this paper is used to evaluate the technological innovation capabilities of enterprises. Standardized data is input from the input layer, and the output data is generated by the system. From this, the level distribution of technological innovation capabilities of the 120 technology-based small and medium-sized enterprises surveyed can be obtained, as shown in Figure 6.

### 4.4. Problems Existing in Enterprise Technological Innovation

Through investigation, it is found that the following problems mainly exist in the process of independent innovation of enterprises. (1) The investment in technological innovation of enterprises is generally low, and the investment structure is unreasonable. The total investment of enterprises in technological innovation is generally low, and they do not pay enough attention to technological innovation, especially lack of long-term strategic planning, and focus on short-term practical results, which is manifested by low investment level and slow growth. (2) Financing is difficult and financing channels are relatively simple. Among the enterprises surveyed, 57.14% of the total accumulated value brought by the policy was in the range of 0 to 1 million; 66.07% of the enterprises received financial subsidies below 1 million; 48.21% of the enterprises did not receive loans from financial institutions. (3) Lack of talents, especially high-level innovative talents. The survey shows that 55.36% of enterprises have fewer than 50 scientific and technical personnel. From the perspective of the structure of scientific and technical personnel, there is a lack of participation of highly educated employees at the level of doctoral and master's degrees, and the lack of support from high-level titles and high-quality talents. This situation is particularly prominent in companies with severely insufficient technological innovation capabilities. (4) Difficulties in market information. Without the support of information technology and information systems, enterprises wanting to engage in technological innovation is tantamount to working behind closed doors. Insufficient information system support for technological innovation. Among the companies surveyed, 33.93% of the companies do not have an information resource database, and 32.14% of the companies do not have an information system. Naturally, it is difficult for these companies to obtain technical information and market information. Without the support of information technology and information systems, enterprises wanting to engage in technological innovation is tantamount to working behind closed doors. (5) Technological innovation has not been paid attention to in the overall strategy of the enterprise. The survey shows that 46.42% of companies have a clear understanding of the company's own mission, vision, business philosophy, corporate spirit, and strategy, and at the same time it also reflects the important position of innovation in corporate strategy. However, 53.58% of companies do not realize the importance of innovation in the overall strategy.

The article "Research on the Evaluation Method of Enterprises' Independent Innovation Ability Based on Improved BP Neural Network and DQN Algorithm" was retracted in 2023. Reasons: unreliable results or conclusions; concerns about the data; concerns about the results or conclusions; concerns about the peer review.

### 4.5. Countermeasures

This article proposes the following countermeasures for the aforementioned problems. (1) Enhance corporate innovation awareness and increase investment in technological innovation resources. (2) Adjust the investment structure of technological innovation and rationally allocate resources. (3) Improve internal management mechanisms and broaden corporate financing channels. (4) Establish a talent incentive mechanism, and actively cultivate and introduce technological innovation talents. (5) Accelerate the construction of enterprise informatization and improve the supporting system for technological innovation.

## 5. Conclusions

Science and technology enterprises are an important source of national economic growth, and the seeds and foundations of large-scale high-tech enterprises in the future. How to measure and improve one's own technological innovation capability is particularly important for technological enterprises based on technological innovation. On the basis of relevant literature research and theoretical review, this paper constructs an evaluation index system based on excellent performance, and explains the specific indicators. Conduct empirical research through training samples and test samples to verify the effectiveness of the evaluation model; finally, combined with the specific conditions of the 120 companies surveyed, this paper comprehensively analyzes the characteristics and existing problems of technological innovation in technology-based enterprises, and analyzes the characteristics and existing problems of technological innovation from the enterprises themselves. From the perspective, practical countermeasures, to improve technological innovation are put forward, capacity, and at the same time put forward corresponding policy recommendations from the perspective of the government.

## Figures and Tables

**Figure 1:** The technical roadmap.

**Figure 2:** The structure of BP network.

**Figure 3:** The structure of BP network.

**Figure 4:** Loss drop curve for network training.

**Figure 5:** Error of test sample.

**Figure 6:** Enterprise technology independent innovation capability level distribution.

The article "Research on the Evaluation Method of Enterprises' Independent Innovation Ability Based on Improved BP Neural Network and DQN Algorithm" was retracted in 2023. Reasons: unreliable results or conclusions; concerns about the data; concerns about the results or conclusions; concerns about the peer review.

**Table 1:** Distribution of enterprise technology fields.

Technical field	Quantity	Proportion (%)
Digital information	20	16.7
Biomedicine	15	12.5
New material	30	25
Optoelectronics	44	36.7
New energy	5	4.2
Resource environment	6	5
Service industry	0	0
Platform project	0	0
Total	120	100

## Data Availability

The data used to support the findings of this study are available from the corresponding author upon request.
